# LncRNA PVT1 Promotes Hypoxia-Induced Cardiomyocyte Injury by Inhibiting miR-214-3p

This article has been retracted.

**DOI:** 10.1155/2021/4604883

**Published:** 2021-11-15

**Authors:** Chuanliang Liu, Jieqiong Zhang, Xuejie Lun, Lei Li

**Affiliations:** ^1^The First Department of Health Care, Weifang People's Hospital, China; ^2^The Third Department of Health Care of Weifang People's Hospital, 151 Guangwen Street, Kuiwen District, Weifang City, 261041 Shandong Province, China; ^3^Department of Internal Medicine, Weifang Municipal Hospital, China

## Abstract

**Objective:**

To explore the effect and related mechanism of LncRNA PVT1 on hypoxia-induced cardiomyocyte injury.

**Methods:**

PVT1RNA and miR-214-3p levels were detected by quantitative real-time polymerase chain reaction (qRT-PCR). Cell vitality and apoptosis were, respectively, evaluated by Cell Counting Kit-8 (CCK-8) and flow cytometry analysis. Starbase and Dual luciferase reporter (DLR) gene assay was employed to validate the interaction between miR-214-3p and PVT1.

**Results:**

PVT1 was statistically upregulated, and miR-214-3p was statistically downregulated in hypoxia-induced H9c2 cells. The survival rate of H9c2 cells induced by hypoxia decreased statistically, while the apoptosis rate increased statistically (*P* < 0.05). PVT1 knockdown upregulated the hypoxia-induced H9c2 cell viability and inhibited apoptosis. DLR assay verified the targeting relationship between PVT1 and miR-214-3p. In addition, miR-214-3p inhibitors reversed the viability of H9c2 cells with PVT1 knockout and promoted apoptosis.

**Conclusion:**

Silencing PVT1 can enhance the hypoxia-induced H9c2 cell viability and inhibit apoptosis, providing a potential target for the treatment of cardiovascular diseases.

## 1. Introduction

As a common disease, the incidence of cardiovascular diseases (CVDs) keeps increasing as the social environment and living habits change, which hazards human life safety [1, 2]. Today, along with the advances in science and technology and the development of medical technology, people's understanding of CVDs is also constantly making breakthroughs [3]. While for CVDs, it is of the essence to explore the mechanism of its occurrence and development and to find effective therapeutic drugs or targets.

In CVDs, cardiomyocyte injury is among the key factors leading to the occurrence and development of the disease [4]. For example, in acute myocardial infarction, myocardial ischemia/reperfusion is among the most pervasive types of myocardial injury in clinical practice [5]. Previous studies [6] have pointed out that cardiomyocyte apoptosis is the main form of cardiomyocyte injury; so, exploring the mechanism of cardiomyocyte apoptosis and how to prevent it is vital for the treatment of CVDs patients. LncRNA, as a noncoding long strand RNA, plays a biological role in cells mainly through regulating protein transcription and has been found to be essential in a wide spectrum of diseases in recent years, including CVDs [7]. For example, a study [8] found that inhibition of lncRNA MALAT1 statistically increased miR-558, decreased the survival rate, and increased the apoptosis rate of isoproterenol-treated H9c2 cells. LncRNA PVT1 is an oncogene that exerts marked effects on multiple tumors, and studies in recent years have found that it also plays a key role in some CVDs [9, 10]. For instance, a study [11] found that lncRNA PVT1 was statistically increased in cardiac tissues of mice with cardiac hypertrophy. However, up to now, the mechanism of PVT1 in cardiomyocyte injury remains poorly understood.

Therefore, through the establishment of cardiomyocyte injury model, we inquired into the effect of lncRNA PVT1 on cardiomyocyte injury and its related mechanism, in order to provide more target directions for CVD prevention and treatment.

## 2. Materials and Methods

### 2.1. Culture and Modeling of Cells

At 37°C, cardiomyocyte H9c2 cells (Shanghai Cell Bank of Chinese Academy of Sciences) were placed in DMEM (Dulbecco's Modified Eagle Medium; Thermo Fisher Science, Inc., Waltham, MA, USA) with 10% FBS (fetal bovine serum; Gibco, Gran Island, NY, USA) and 100 *μ*g/mL penicillin/streptomycin (Invitrogen, Thermo Fisher Scientific) and 5%CO_2_ for incubation. Then, the cardiomyocytes were collected for transfection when the adherent growth reached 80% and classified into the hypoxia group and control group. In the hypoxia group, H9c2 cells were cultured with a mixture of 1% O_2_, 94% N_2,_ and 5% CO_2_ within a specified time, and those in control group shared the same culture conditions besides that the O_2_ concentration was 21%.

### 2.2. Transfection of Cells

As to the small interfering RNAs (si-PVT1-#1, si-PVT1-#2, si-PVT1-#3) and the control siRNA (si-NC) of PVT1, they were all obtained from Shanghai GenePharma (Shanghai, China). MiR-214-3p mimic sequence (miR-214-3p-mimics), miR-214-3p targeted inhibition sequence (miR-214-3p-inhibitor), and miR negative control (miR-NC) were constructed by FitGene Co., Ltd. (Guangzhou, Guangdong, China). Strictly following the manufacturer's instructions, cells' transfection was performed with Lipofectamine™ 2000 kit (Invitgen, Carlsbad, CA, USA).

### 2.3. qRT-PCR

From tissues and cells, total RNA was separated with the aid of Trizol Reagent, and 5 *μ*g of it was subjected to reverse transcriptional cDNA as instructed by the instructions. Finishing transcription, synthetic cDNA (1 *μ*L) was processed for amplification. PCR reaction conditions (40 cycles) are as follows: 60 s predenaturation at 95°C, 40 s denaturation at 95°C, and 40 s extension anneal at 60°C. MiR-214-3p used U6 as a control, PVT1 used GAPDH as an internal reference, and 2^-△△ct^ was responsible for data analysis. See Table 1 for primer sequences.

### 2.4. Cell Proliferation Test

H9c2 cell viability was evaluated by CCK-8. 48 h after transfection, the cells were diluted to 3 × 10^5^cells/mL and inoculated into 96-well plates (3000 cells/well) with 100 *μ*L cells per well for culture in normal or hypoxic medium. Then, at 48 hours of culture, 10 *μ*L CCK8 solution (10 *μ*L, Sigma, SF, USA) was added for another 2 h of culture in the incubator at 37°C and 5% CO_2_. With the aid of a microplate reader (Bio-Rad, Cal, USA), OD value at 450 nm was measured for cell proliferation determination and growth curve plotting. The experiment was conducted in triplicate.

### 2.5. Apoptosis Test

Finishing digestion with 0.25% trypsin, the cells were rinsed with PBS twice, immersed in binding buffer (100 *μ*L) to rearrange to 1 × 10^6^ cells/mL, and added with Annexin V-FITC and PI with 10 *μ*L each successively for 5-minute culture at indoor temperature in dark place. Flow cytometry system was used for detection, and the experiment was conducted in triplicate to average the value.

### 2.6. Western Blotting

The total protein of HUVEC was obtained by using a RIPA lysis buffer (Cell Signal Technology, Danvers, MA, USA) containing protease inhibitors. The proteins were then separated by SDS-PAGE (10%) with sodium dodecyl sulfate-polyacrylamide gel electrophoresis and transferred to a PVDF membrane (MilliPore, Bilerika, Ma, USA). After sealing with 5% skimmed milk and TBST, it was cultivated all night long at 4°C with anti-Bcl-2 (1 : 500), Bax (1 : 500), cle-caspase-3 (1 : 500), or GAPDH(1 : 1000) (Abcam, Cambridge, Massachusetts, USA). Then, at indoor temperature, it was immersed in horseradish peroxidase-labeled goat anti-rabbit secondary antibody (1 : 1000; Wuhan Boster Biological Technology Co., Ltd.) for 1-hour culture, followed by 3 times of rinsing with PBS, 5 min each. In a dark room, development was carried out under the prerequisite that the excess liquid on the film was blotted with a filter paper and then illuminated by ECL to develop.

### 2.7. DLR Assay

The potential miRNAs that could bind to PVT1 was screened through the bioinformatics database starBase v2.0. Oligonucleotides containing PVT1 target sequences were then amplified and cloned into pmirGLO plasmid (WT). The wild type (Wt) and mutant (Mut) of pmirGLO-PVT1-3′UTR were established, respectively, and transferred to the downstream of the luciferase reporter gene for sequencing and identification of the constructed plasmids. By referring to the manufacturer's instructions, Lipofectamine 2000 (Invitrogen, Thermo Fisher Scientific, USA) was used to cotransfect the plasmids constructed above with miR-214-3p-mimcs and miR-NC into H9c2 cells. The luciferase activity after 48 hours of incubation was determined by dual luciferase assay system.

### 2.8. RIP Detection

As instructed by the guidelines, EZ-Magna RIP kit (Shanghai Advantage Biological Co., Ltd.) was utilized for RNA immunoprecipitation. From the culture plate, H9c2 cells were scraped and lysed in 100% RIP Lysis Buffer. Then, the cell extracts were left in the RIP buffer supplemented with magnetic beads, which could adsorb human anti-AGO2 antibody (1 : 2000, Abcam, USA). Finally, protease K was used for sample digestion and RNA extraction for WB analysis. Immunoglobulin G (IgG) (1 : 1000, Abcam, USA) was used as a negative control. Acquired from Thermo Fisher Scientific, NanoDrop spectrophotometer was used to detect RNA concentration, while RNA quality was analyzed by a Bioanalyzer obtained from Agilent Corporation, Santa Clara, California, USA. The experimental samples were repeated three times.

### 2.9. RNA Pull-down Assay

Biotin-labeled PVT1 (1 *μ*g) was loaded into the Eppendorf (EP) test tube using magnetic RNA protein pull-down kit (Pierce, Rockford, IL, USA). Then, structural buffer was added for a 2-minute bath at 95°C and a 3-minute ice bath successively. After incubating 50 *μ*L fully resuspended beads overnight in EP tube at 4°C, the beads were centrifuged at the speed of 1500 × g for 3 minutes to discard the supernatant and then rinsed with 500 *μ*L RNA binding protein immunoprecipitation (RIP) washing solution for 3 times. After washing, they were added with 10 *μ*L cell lysis buffer and left to stand for 1 h at indoor temperature. At low speed, the cultured bead-RNA-protein mixture was centrifuged, and the obtained supernatant was rinsed with 500 *μ*L RIP washing buffer for three times after centrifugation. Finally, taking 10 *μ*L cell lysate supernatant as the input protein, the protein expression profiles were determined by WB. The experiment was carried out in triplicate.

### 2.10. Statistical Processing

SPSS19.0 and GraphPad 7 were employed for analysis and image rendering of the experimental data, respectively. Comparison between groups was performed by independent *t*-test, those among multiple groups were done by one-way ANOVA, and postpairwise comparisons were done by LSD-t. Multitime expression profiles were analyzed by repeated measures ANOVA, and posthoc tests were conducted by Bonferroni. *P* < 0.05 indicated a statistically significant difference.

## 3. Results

### 3.1. Hypoxia Induced PVT1 Upregulation in Cardiomyocyte H9c2 Cells

When we established a model of H9c2 cell injury using hypoxia induction, PVT1 was found to be enhanced, and miR-214-3p was statistically declined in H9c2. The effect of hypoxia induction was evaluated by measuring the cell survival rate and the proportion of apoptotic cells. The survival rate of H9c2 cells was statistically reduced, and the apoptosis rate was statistically increased after hypoxia compared with control group. We further found that in hypoxia-induced H9c2 cells, apoptotic proteins Bax and CLE-Caspade-3 increased, while antiapoptotic protein Bcl-2 decreased. It is suggested that PVT1 may be related to H9c2 cell damage induced by hypoxia (Figure 1).

### 3.2. Knocking Down PVT1 Attenuated Hypoxia-Induced Cardiomyocyte Injury

Si-PVT1 was used to downregulate PVT1 to study PVT1's role in hypoxia-induced injury of H9c2 cells. According to transfection efficiency, the inhibition efficiency of si-PVT1-#1 transfection was the highest. Downregulation of PVT1 evidently lowered hypoxia-induced cell injury through increasing cell survival rate and reducing apoptosis rate. In addition, PVT1 downregulation suppressed apoptotic proteins Bax and cle-caspase-3 and elevated Bcl-2. It shows that downregulation of PVT1 can reduce hypoxic-induced cardiomyocyte injury (Figure 2).

### 3.3. PVT1 Could Sponge miR-214-3p

With the aim of further exploring the mechanism of the action of PVT1 on H9c2 cells, we predicted the potential miRs of PVT1 through starbase online and found that there were potential binding targets between PVT1 and miR-214-3p, which were further verified by DLR, RIP test, and pull-down test. The dual luciferase reporter assay revealed miR-214-3p-mimics markedly suppressed PVT1-WT fluorescence activity. RIP assay identified that PVT1 and miR-214-3p levels precipitated by Ago2 antibody were statistically increased compared with IgG (Figure 3).

### 3.4. PVT1 Sponge Adsorption of miR-214-3p Aggravated Hypoxia-Induced Cardiomyocyte Injury

With the purpose of confirming whether PVT1 affected hypoxia-induced cardiotoxicity through sponge adsorption of miR-214-3p, we transfected miR-214-3p inhibitor into H9c2 cells and found that miR-214-3p was statistically inhibited. MiR-214-3p inhibitor statistically decreased the viability of H9c2 cells with PVT1 knockout and promoted apoptosis after cotransfecting miR-214-3p inhibitor plus Si-PVT1 into hypoxia-induced H9c2 cells. Similarly, miR-214-3p inhibitors downregulated Bcl-2 and promoted Bax and cle-caspase-3. It suggests that by sponging miR-214-3p, PVT1 aggravates hypoxia-induced cardiomyocyte injury. (Figure 4).

## 4. Discussion

The pathomechanism of CVD is a complex and multifactorial process. The primary mechanism of CVD is atherosclerosis. Inflammation in atherogenesis raises the risk of hypoxia, which will activate hypoxia-inducible factor-1*α* (HIF1A) [12, 13]. Tissue hypoxia seems to be one of the common features in cardiovascular disorders including atherosclerosis, vascular remodeling, and heart failure. In the hypoxic environment, each cell exhibits several types of responses at transcriptional, translational, or posttranslational levels. Most of the gene expressions are, at the transcriptional level, significantly suppressed in the hypoxic environment. In contrast, the expression of a group of genes is significantly enhanced in hypoxia, including hypoxia-inducible genes [12]. At present, how to improve hypoxia-induced cardiomyocyte injury is also a hot research direction. It has been proposed that some intracellular proteins, such as protein kinase [14] and heat stress protein [15], can be used to provide endogenous myocardial protection against hypoxia induced cardiomyocyte injury, whereas clinically understanding the mechanism of hypoxic cardiomyocytes injury is of the essence for the treatment of CVDs.

LncRNA, as a popular noncoding RNA in recent years, has also been extensively studied in the treatment of CVDs [16]. For example, a study [17] found that inhibiting lncRNA NEAT1 could reduce hypoxia-induced cardiomyocyte injury through sponging miR-378a-3p. However, few studies have investigated the role and mechanism of lncRNA PVT1 in hypoxic cardiomyocyte injury. In our study, we first observed a significant decrease in survival rate of hypoxic-induced cardiomyocytes and a significant increase in apoptosis rate, suggesting that PVT1 may be related to hypoxia-induced cardiomyocyte injury. In the study of Sun et al. [18], PVT1 was highly expressed in patients with heart failure, which was in line with our results. Then, for the purpose of further analyzing PVT1's effect on hypoxia-induced cardiomyocytes, we knocked down PVT1. The results showed that when PVT1 in hypoxia-induced injury cardiomyocytes was knocked down, the cell survival rate was statistically improved, and the apoptosis rate was statistically decreased, suggesting that the injury of cardiomyocytes was improved. Currently, the role of PTV1 in hypoxia-induced cardiomyocyte injury has not been explored. Although here we have found for the first time that inhibition of PTV1 can improve hypoxia-induced cardiomyocyte injury, the specific downstream mechanism remains unknown.

It is well known that LncRNA may play a role of molecular sponge in regulating miRNA expression and biological function [19]. This also provides new insights into exploring the downstream molecular mechanism of PVT1 on hypoxia-induced cardiomyocyte injury. Increasing evidence has confirmed the role of miRNAs in CVDs. Zhang et al. [20] revealed that miR-27 reduced hypoxia/reoxygenation induced cardiomyocyte injury by targeting TGFBR1 and inhibiting NF-*κ*B pathway. Ma et al. [21] found that by targeting PDCD4, miR-532-5p could reduce hypoxia-induced cardiomyocyte apoptosis. Subsequently, we found through the prediction of biological information that there were shared sites between PTV1 and miR-214-3p. It is reported [22] that the lack of miR-214-3p aggravates cardiac fibrosis. There is also evidence [23] showing that miR-214-3p is linked with cardiomyocyte apoptosis in diabetic cardiomyopathy. In our study, miR-214-3p declined statistically in hypoxia-induced cardiomyocytes, and subsequently, DLR, RIP, and pull-down experiments verified that PVT1 can directly bind miR-214-3p, which suggested that PVT1 played its role in hypoxia-induced cardiomyocyte injury through sponging miR-214-3p. Finally, to further prove the targeting effect of PVT1 on miR-214-3p, cotransfection of miR-214-3p inhibitor and Si-PVT1 was conducted on hypoxia-induced H9c2 cells. It was observed that miR-214-3p inhibitor statistically inhibited the viability of PVT1 knock-out H9c2 cells and promoted apoptosis, which further proved that PVT1 could affect hypoxia-induced cardiomyocyte by through sponging miR-214-3p.

Recently, the crosstalk between miRNAs and long noncoding RNA (lncRNA) has attracted increasing attention leading to the identification of new regulatory networks (reviewed by Ballantyne et al. and Yoon et al. [24]). An example of such crosstalk is the interaction between lncRNA MiR143HG and miR-143/145: the focus of this review. Mir-143/145 is a vascular-enriched miRNA cluster, fairly extensively studied in vascular biology and in the pathophysiology of cardiovascular disease [25–30]. This microRNA cluster was shown to be encoded in a bicistronic unit [30] located downstream of the lncRNA MiR143HG, host gene of the miR-143 miRNA. Notably, the structure, the expression, and the function of lncRNAs have gained increasing attention, resulting in rapid progression in the understanding of their potential importance.

In addition, previous findings suggested that silencing of PVT1 improved spatial learning and memory, decreased neuronal loss, the number of TUNEL-positive cell, and the expression of cleaved-caspase-3 and Bax while increased the procaspase-3 and Bcl-2 expression in hippocampus tissues in epileptic rats. Furthermore, silencing of PVT1 decreased the expression of axin and cyclin D1 in hippocampus tissues in epileptic rats [31].

In summary, lncRNA PVT1 can play a role in hypoxia-induced cardiomyocyte injury by sponging miR-214-3p, which is a feasible biological biomarker for diagnosing and treating CVDs. However, our study is limited by the small sample size. In addition, the function of PVT1 in CKD and the molecular mechanism remain unclear. Further study is necessary to find the optimal hypoxic pattern of different cell types. Understanding the mechanism of lncRNA PVT1 would undoubtedly provide important insight into its role in CVDs and provide potential approaches to regulate its expression, including sirRNA or gene editing.

## Figures and Tables

**Figure 1:** Hypoxia induced PVT1 upregulation in cardiomyocyte H9c2 cells. (a) PVT1 and miR-214-3p expression in H9c2 cells induced by hypoxia. (b) Survival rate of H9c2 cells induced by hypoxia. (c) Apoptosis rate of H9c2 cells induced by hypoxia. (d) Expression of apoptosis-related proteins in H9c2 cells induced by hypoxia. ^∗^ indicated *P* < 0.05.

**Figure 2:** Knockdown of PVT1 alleviated hypoxia-induced cardiomyocyte injury. (a) Knockdown efficiency of PVT1 in cardiomyocytes. (b) Effects of PVT1 knockdown on the survival rate of hypoxic-induced cardiomyocytes. (c) Effects of PVT1 knockdown on the apoptosis rate of hypoxic-induced cardiomyocytes. (d) Effects of PVT1 knockdown on apoptosis-related proteins in hypoxic-induced cardiomyocytes. ^∗^ indicated *P* < 0.05.

**Figure 3:** Relationship between PVT1 and miR-214-3p. (a) DLR confirmed that there was a binding relationship between PVT1 and miR-214-3p. (b) Enrichment ability of PVT1 and AGO2 evaluated by RIP assay. (c) Enrichment ability of PVT1 and miR-214-3p determined by RNA pull-down. ^∗^ indicated *P* < 0.05.

**Figure 4:** PVT1 sponge adsorption of miR-214-3p aggravated hypoxia-induced cardiomyocyte injury. (a) Inhibition efficiency of miR-214-3p in cardiomyocytes. (b) Effects of cotransfection of miR-214-3p-inhibitor and Si-PVT1 on viability of cardiomyocytes induced by hypoxia. (c) Effects of cotransfection of miR-214-3p-inhibitor and Si-PVT1 on the apoptosis rate of cardiomyocytes induced by hypoxia. (d) Effects of cotransfection of miR-214-3p-inhibitor and Si-PVT1 on apoptosis-related proteins in cardiomyocytes induced by hypoxia. ^∗^ indicated *P* < 0.05.

**Table 1:** Primer sequences.

Gene	Upstream primer (5′-3′)	Downstream primer (5′-3′)
miR-214-3p	ACAGCAGGCACAGACAGG	GTGCAGGGTCCGAGGT
U6	AAAATTTCTCACGCCGGTATTC	CCTGCAGACCGTTCGTCAA
PVT1	GCCCCTTCTATGGGAATCACTA	GGGGCAGAGATGAAATCGTAAT
GAPDH	GGAGCGAGATCCCTCCAAAA	GGCTGTTGTCATACTTCTCATGG

## Data Availability

The authors confirm that the data supporting the findings of this study are available within the article.
